RETRACTED

# Electrospun Ta-MOF/PEBA Nanohybrids and Their CH_4_ Adsorption Application

**DOI:** 10.3389/fchem.2022.868794

**Published:** 2022-06-16

**Authors:** Saade Abdalkareem Jasim, Jihad M. Hadi, Abduladheem Turki Jalil, Maria Jade Catalan Opulencia, Ali Thaeer Hammid, Mohadeseh Tohidimoghadam, Mohammadreza Moghaddam-manesh

**Affiliations:** ^1^ Medical Laboratory Techniques Department, Al-Maarif University College, Ramadi, Iraq; ^2^ Department of Medical Laboratory of Science, College of Health Sciences, University of Human Development, Kurdistan Regional Government, Slemani, Iraq; ^3^ Medical Laboratories Techniques Department, Al-Mustaqbal University College, Hilla, Iraq; ^4^ College of Business Administration, Ajman University, Ajman, United Arab Emirates; ^5^ Computer Engineering Techniques Department, Faculty of Information Technology, Imam Ja’afar Al-Sadiq University, Baghdad, Iraq; ^6^ Pasteur Hospital, Bam University of Medical Science, Bam, Iran; ^7^ Petrochemistry and Polymer Research Group, Chemistry and Petrochemistry Research Center, Standard Research Institute, Karaj, Iran

**Keywords:** Ta-MOF/PEBA, ultrasonic-assisted electrospinning, CH_4_ adsorption, fibrous polymer, air pollution

## Abstract

For the first time, biocompatible and biodegradable Ta-metal organic framework (MOF)/polyether block amide (PEBA) fibrous polymeric nanostructures were synthesized by ultrasonic and electrospinning routes in this study. The XRD peaks of products were wider, which is due to the significant effect of the ultrasonic and electrospinning methods on the final product. The adsorption/desorption behavior of the nanostructures is similar to that of the third type of isotherm series, which showed mesoporous behavior for the products. The sample has uniform morphology without any evidence of agglomeration. Since the adsorption and trapping of gaseous pollutants are very important, the application of the final Ta-MOF/PEBA fibrous polymeric nanostructures was investigated for CH_4_ adsorption. In order to achieve the optimal conditions of experiments and also systematic studies of the parameters, fractional factorial design was used. The results showed that by selecting temperature 40°C, time duration 35 min, and pressure 3 bar, the CH_4_ gas adsorption rate was near 4 mmol/g. Ultrasonic and electrospinning routes as well as immobilization of Ta-MOF in the PEBA fibrous network affect the performance of the final products for CH_4_ gas adsorption.

## 1 Introduction

In recent years, due to the expansion of industries, gaseous pollutants have increased significantly (Zheng et al., 2018). The effects of these pollutants have become so severe that reducing them has attracted the attention of communities and organizations (Afroz et al., 2003). One of the gas pollutants that has adverse effects on the environment, plants, and animals is CH_4_ (Van Amstel, 2012). Due to its harmful momentary effects, trapping CH_4_ using a desirable device is very important and critical (Murseli et al., 2019).

RETRACTED

In the last few years, different nanostructures such as active carbon and zeolite have been studied in the field of CH_4_ gas adsorption due to their desirable potential properties (Rios et al., 2013; Mofarahi and Gholipour, 2014). Recently, metal organic frameworks (MOFs) have been used for the adsorption of CH_4_ gas pollution due to their high specific surface area, stable chemical properties, high thermal stability, and significant porosity (Szczęśniak et al., 2018; Wu et al., 2019). Although the efficiency of these samples for trapping CH_4_ is desirable, increasing their surface area properties for surface interaction between MOF nanostructures and CH_4_ molecules is very important (Wang et al., 2018).

On the other hand, the use of biocompatible and biodegradable fibrous polymers has recently received attention. These compounds with various capabilities in the fields of medicine, engineering, and environment, depending on their properties, have various functions (Zhou et al., 2021; Hu et al., 2022; Li et al., 2022).

Fibrous nanostructures can be synthesized in various methods, and one of the most effective routes is electrospinning. This technique is rapidly developing from the single-fluid blending process (Li et al., 2021a; Homaeigohar and Boccaccini, 2022) to coaxial (Sapountzi et al., 2020; He et al., 2021a), side-by-side (Li et al., 2021b), tri-axial (Wang et al., 2020) and other complicated processes (He et al., 2021b; Luo et al., 2021). These processes expand the capabilities of electrospinning in creating novel functional nanomaterials by encapsulating different kinds of functional ingredients, including nanoparticles (Xue et al., 2021; Zhang et al., 2022).

If MOF nanostructures are integrated with fibrous polymers, their properties are expected to increase in particular, which will affect the performance of the samples (Sargazi et al., 2020). On the other hand, this also affects the specific surface of the final products, which results in the creation of compounds with high tendencies in the interaction between the surface of the structure and gas (Wang et al., 2019).

Systematic design of parameters in order to achieve maximum gas adsorption is very important. In non-systematic methods, the interaction between experimental parameters such as temperature, time duration, and pressure is not considered. In addition, achieving the optimal amount of CH_4_ gas adsorption without considering the interaction between experimental parameters (temperature, time duration, and pressure) is a problem. Therefore, examining the effect of experimental parameters on CH_4_ gas adsorption is a deep challenge (Pu et al., 2021).

RETRACTED

In this study, for the first time, Ta-MOF/PEBA fibrous polymer nanostructures were synthesized by ultrasonic and electrospinning procedures. The resulting nanostructures were characterized by scanning electron microscopy (SEM) with energy-dispersive spectroscopy (EDS), thermogravimetric analysis (TGA), Brunauer–Emmett–Teller (BET) technique, and Fourier transform infrared spectroscopy (FT-IR). The resulting samples are used as a novel option for CH_4_ gas adsorption. In order to deeply understand the amount of temperature, time duration, and pressure on CH_4_ adsorption, a fractional factorial design has been used.

## 2 Experimental Section

### 2.1 Material Characterization

Ta (NO_3_)_5_.6H_2_O, poly ether black amide (PEBA), and acetic acid were purchased from Sigma-Aldrich. All these chemicals were of analytical grade and were used without further purification. The microstructure behaviors of Ta-MOF/PEBA fibrous nanostructure samples were investigated by a scanning electron microscope (SEM, JEOL JSM6700F). Fourier transform infrared spectra (FT-IR, Nicolet IS10 IR spectrophotometer) were applied to characterize the related groups in the final structures.

The crystal behavior of the products was recorded by using a Scintag X1 diffractometer with monochromatized Cu–Kα irradiation (*λ* = 0.1540 nm) to recognize X-ray diffraction patterns. BET surface areas of Ta-MOF were investigated by a Micromeritics TriStar II 3020, Norcross, GA, gas adsorption analyzer. Thermogravimetric behaviors of the products were characterized by a DuPont TA Q50 analyzer.

### 2.2 Synthesis of Ta-MOF Nanostructures

In an ultrasonic typical synthesis, 2 mg of Ta (NO3)_5_.6H_2_O and 6 mg of pyridine-2,6 dicarboxylic acid were dissolved in 50 ml of acetic acid. The resulting solution was placed in a magnetic stirrer for 40 min at 70°C. The mixture was transferred to an ultrasonic bath and irradiated under optimal ultrasonic conditions including temperature: 30°C, power: 150 W, and irradiation time: 70 min. Finally, white crystals of Ta-MOF were obtained after calcination under an argon atmosphere at 160°C.

### 2.3 Synthesis of Ta-MOF/PEBA Fibrous Polymeric Nanostructures

In order to synthesize Ta-MOF/PEBA fibrous polymeric nanostructures, the Ta-MOF nanostructures synthesized in the previous step (section 2.2) were dissolved in 25 ml of acetic acid. The final solution was homogenous under a magnetic stirrer at 150°C. The mixture was transferred into an electrospinning device at flow rate: 0.2 ml/h, voltage: 27 KV, PEBA concentration: 40 wt%, and spinning distance: 50 cm. Finally, the Ta-MOF/PEBA fibrous polymeric product was calcined at 180°C under an argon atmosphere.

RETRACTED

### 2.4 CH_4_ Gas Adsorption

To investigate CH_4_ gas adsorption by Ta-MOF/PEBA fibrous polymeric nanostructures, a setup according to a voltametric method was used. The purity of CH_4_ in the gas reactor was increased to 90% by the first generation of the GAMA PURIFICATION unit. The details of gas adsorption were reported in the previous work (Sargazi et al., 2020). The process was such that, first, a valve was installed between the dozer (storage reservoir) and tank (adsorption reservoir). Consequently, the number of CH_4_ gas moles in the dozer was calculated using Eq. 1:

$${\text{P}}_{1}{\text{V}}_{1}{=\text{Z}}_{1}{\text{N}}_{1}\text{RT }\Rightarrow N1=\frac{P1V1}{\text{Z}1\text{RT}},$$ (1)

where P_1_, N_1_, R, T, and Z_1_ show gas pressure, number of gas moles, general constant of gases, equilibrium temperature, and compressibility coefficient in the dozer, respectively. In the second step, the valve between the two reservoirs was opened and the Ta-MOF/PEBA fibrous products were placed inside the tank. Thus, as a result of transmission of gases into the tank, the amount of the CH_4_ gas moles in tank could be calculated by Eq. 2:

$${\text{P}}_{2}{\text{V}}_{2}{=\text{Z}}_{2}{\text{N}}_{2}\text{RT }\Rightarrow N2=\frac{P2V2}{\text{Z}2\text{RT}},$$ (2)

where P_2_, Z_2_, and V_2_ presented gas pressure, compressibility coefficient factor in the adsorption reservoir, and total volume of the adsorption and storage reservoirs, respectively. Finally, the gas moles adsorbed by the Ta-MOF/PEBA electrospun nanofibrous composite could be calculated by n_ADS_= n_1_-n_2_.

## 3 Result and Discussion

### 3.1 Physico-Chemical Properties

XRD patterns of Ta-MOF/PEBA fibrous polymeric network are shown in Figure 1A. The existence of broad peaks in the final structures confirmed the nano-structural nature of these compounds. It can be related to the effective effect of ultrasonic and electrospinning routes on the final product (Sargazi et al., 2018).

**FIGURE 1:** XRD patterns in 2 theta angle of 0–90 **(A)**, TG curve in the range of 0–700°C **(B)**, N_2_ adsorption/desorption behavior, **(C)** and BJH plot **(D)** for Ta-MOF/PEBA fibrous polymer.

Figure 1B shows the thermal stability of the Ta-MOF sample immobilized on the PEBA fibrous polymeric network from room temperature up to 600°C in order to study the thermal properties of the samples.

According to TG analysis, the main weight losses observed at 342°C can be attributed to the decomposition of frameworks in the network. As an important result, the Ta-MOF/PEBA fibrous polymeric sample has high thermal stability up to 340°C. It seems that the product developed in this study has more thermal stability than the pure Ta-MOF sample synthesized in the previous sample (Sargazi et al., 2018). Higher thermal stability of the electrospun products can be attributed to the incorporating physiochemical properties of the Ta-MOF and PEBA fibrous network. The synthesis of samples with high thermal stability provides the capability of final products in different areas.

RETRACTED

The adsorption/desorption isotherm of the Ta/PEBA fibrous polymeric network samples is shown in Figure 1C. The adsorption/desorption behavior of this sample is similar to the third type of isotherm series, which showed mesoporous behavior for the products (Ebadi et al., 2009). According to the BET technique, the specific surface area of the sample is about 3700 m^2^/g, which is significantly increased compared to the pure Ta-MOF sample (1784 m^2^/g) (Sargazi et al., 2018). It seems that the participation of samples in fibrous networks and the effective effects of ultrasonic and electrospinning routes have significantly affected the specific surface area and porosity of the Ta-MOF/PEBA fibrous network. Figure 1D also showed the pore size distribution of the final products obtained by the BJH method. According to this method, Ta-MOF/PEBA fibrous nanostructures have mesoporous size distribution with a pore volume of 0.008 cm^3^/g, which is in compliance with the data obtained from N_2_ adsorption/desorption isotherms, while the pure Ta-MOF has a pore volume near 0.002 cm^3^/g.

### 3.2 Morphology With Elemental Mapping

The microstructure results and morphology of the Ta-MOF/fibrous polymeric network are exhibited in Figure 2. As shown in this fig., the nanoparticles are well-immobilized in the network structure, which indicates effective combining of the Ta-MOF and fibrous structures. Also, the morphology of the samples is uniform, which confirms the effective effects of the synthesis route (Bai et al., 2021a; Bai et al., 2021b; Wang et al., 2021). EDS elemental analysis showed the distribution of related elements of Ta-MOF/PEBA nanostructures in the fibrous network. Also, this elemental mapping confirmed the homogenous distribution of samples in the final structures.

**FIGURE 2:** SEM image with EDS elemental analysis of Ta-MOF/PEBA fibrous nanostructures.

### 3.3 Proposed Structures of Ta-MOF/PEBA

Figure 3 shows the FT-IR spectra of Ta-MOF, PEBA, and Ta-MOF/PEBA fibrous nanostructures. In Ta-MOF and PEBA, the presence of a frequency close to 3500 cm^−1^ confirms the NH bonds related to the amine group in the structure (Tang et al., 2020). Also, the presence of bands at 2800 to 3050 cm^−1^ is attributed to the CH aromatic groups in the structures (Hu et al., 2021; Liu et al., 2022). In addition, absorption peaks in the range of 2000 cm^−1^ confirm the presence of various carbonyl groups in the structure. Due to the FT-IR spectrum of Ta-MOF/PEBA, all peaks related to the Ta-MOF and PEBA are observed in the final structure, which is a strong evidence for the successful synthesis of Ta-MOF/PEBA fibrous nanostructures. Also, CHNS/O elemental analysis of Ta-MOF/PEBA is presented in Figure 4. According to the data, the presence of related analysis was confirmed in the final structures. Based on FT-IR spectra and also CHNSO elemental analysis, the suggested structure of Figure 5 was proposed for Ta-MOF/PEBA fibrous network nanostructures.

RETRACTED

**FIGURE 3:** FT-IR spectra of Ta-MOF, PEBA, and Ta-MOF/PEBA fibrous nanostructures.

**FIGURE 4:** CHNS/O elemental analysis for Ta-MOF/PEBA fibrous polymeric nanostructures.

**FIGURE 5:** Proposed structure for Ta-MOF/PEBA fibrous polymeric nanostructures.

### 3.4 Systematic Study

In order to systematically study the process and investigate the effects of experimental parameters on CH_4_ gas adsorption, the fractional factorial method has been used (Bruno Siewe et al., 2021). Experimental parameters include time duration (A), temperature (B), and pressure (C). The design of these parameters has been carried out in three levels (−1, 0, and +1). Table 1 shows the arrangement of these parameters at three levels. The experiments under different conditions are presented in Table 2. All experiments were performed by two replications.

**TABLE 1:** Coded and non-coded ranges of the experimental parameters designed based on the fractional factorial method.

Level	Coded level	Uncoded level		
		Time duration (min)	Temperature (°C)	Pressure (bar)
Low	-1	20	20	1
Medium	0	35	40	2
High	+1	50	60	3
$\text{Coded formula}:\frac{x-\frac{x\;\left(\mathrm{high}\right)+x\left(\mathrm{low}\right)}{2}}{\frac{x\left(\mathrm{high}\right)-x\left(\mathrm{low}\right)}{2}}\text{ , x: }-\omega \;\ldots \text{, }-\text{3, }-\text{2, }-1\text{, 0, }1\text{, }2\text{, }3\text{, }\ldots \text{. }+\omega$				

**TABLE 2:** Randomized fractional factorial designs for CH_4_ gas adsorption obtained by Ta-MOF/PEBA electrospun nanofibrous composite.

Runs	Std order	Center Pt	A (min)	B (°C)	C (bar)	REP	Adsorption (mmol/g)
a	9	1	−1	−1	−1	1	0.7
						2	0.6
b	5	1	0	−1	−1	1	1.4
						2	1.5
c	6	1	0	0	+1	1	4.1
						2	4.0
**d**	3	1	−1	+1	0	1	2.1
						2	2.0
e	2	0	0	0	0	1	3.7
						2	3.9

The residual plot of the experiments was used to investigate the scientific dispersion of experiments and their normal distribution (Huo et al., 2022; Jiang et al., 2021). As shown in Figure 6, the positive and negative levels are strong evidence for dispersion of the experiments on a regular basis. As a result, the dispersion of the experiments confirms the scientific distribution of the process (Wu and Hamada, 2011).

RETRACTED

**FIGURE 6:** Residual plot for different parameters of time duration **(A)**, temperature, **(B)** and pressure **(C)**.

The effect of each of the experimental parameters of time duration, temperature, and pressure on the amount of CH_4_ gas adsorption was investigated by analysis of variance (Table 3). As it is clear, temperature with a P_value_ of 0.000 has a significant effect on CH_4_ gas adsorption. The effect of temperature on the adsorption of CH_4_ gas is in accordance with the previous studies (Liu et al., 2020; Ullah et al., 2020). Pressure has also affected the performance of CH_4_ gas adsorption (Xiao et al., 2009; Xu et al., 2021). According to the PV= znRT equation, the Ta-MOF/PEBA fibrous sample has a remarkable adsorption rate at high pressures. Therefore, the performance of Ta-MOF/PEBA fibrous MOF in condition ***c*** is selected as optimal. Time duration also has a significant effect on CH_4_ adsorption. With increasing time duration, more surface area of the nanostructures comes into contact with the gas, resulting in increased efficiency of CH_4_ gas adsorption. Of course, it should also be taken into account that increasing the contact time to a certain extent can affect the amount of gas adsorption (Kirchstetter et al., 2001).

**TABLE 3:** Analysis of variance for CH_4_ gas adsorption experiments by fractional factorial design.

Source	DF	Seq SS	Adj SS	Adj MS	*P*_*value*_
**A**	1	7.3500	3.6038	3.60375	0.000
**B**	1	6.9769	1.4700	1.47000	0.000
**C**	1	2.0503	0.0625	0.0625	0.038
2-way interactions	3	1.1628	1.1628	1.16281	0.000
A*B	1	1.1628	1.1628	1.1628	0.000

The surface plot has been used to investigate the relationship between experimental parameters of time duration (A), temperature (B), and pressure (C) and gas adsorption. As shown in Figure 7, by selecting different number of experimental parameters, desired values of CH_4_ gas adsorption are obtained. This is a significant relationship between the experimental parameters in accordance with the results of Table 2. The counter plot also confirms this correlation for the experimental parameters and theatrical data (Figure 8). As an important result, optimization of the parameters theatrically facilitates the achievement of desirable conditions.

RETRACTED

**FIGURE 7:** Surface plot of CH_4_ gas adsorption (mmol/g) vs. time duration [**(A)**-min], temperature [**(B)**-°C], and pressure [**(C)**-bar]. Data were reported as coded levels.

**FIGURE 8:** Contour plot of CH_4_ gas adsorption (color legend) vs. time duration **(A)**, temperature **(B)**, and pressure **(C)**. Data were reported as uncoded levels.

## Conclusion

In this study, novel samples of Ta-MOF were synthesized under optimal ultrasonic conditions, including temperature: 30°C, power: 150 W, and irradiation time: 70 min. The resulting Ta-MOF samples were immobilized in PEBA fibrous networks by the electrospinning route. The obtained Ta-MOF/PEBA fibrous polymeric samples with desirable physicochemical properties such as significant specific surface area, high thermal stability, and small size distribution were used as novel candidates in the adsorption of gaseous pollutants. Factorial analysis has been used to investigate the effect of experimental parameters on the performance of products and also to systematically study the process. Analysis of variance confirmed the effects of time duration, temperature, and pressure on the efficiency of the Ta-MOF/PEBA fibrous sample in CH_4_ gas adsorption. The compounds synthesized in this study open a new window to introduce effective biocompatible and biodegradable compounds for developing other gaseous pollutants.

## Data Availability

The original contributions presented in the study are included in the article/Supplementary Materials; further inquiries can be directed to the corresponding author.
